This article has been retracted.

# LCZ696 Ameliorates Isoproterenol-Induced Acute Heart Failure in Rats by Activating the Nrf2 Signaling Pathway

**DOI:** 10.1155/2022/6077429

**Published:** 2022-04-29

**Authors:** Min Hou, Linxin Lu, Xiaobo Wu, Hongxuan Liu

**Affiliations:** ^1^Department of Emergency, Shanxi Bethune Hospital, Shanxi Academy of Medical Sciences Tongji Shanxi Hospital, Third Hospital of Shanxi Medical University, Taiyuan 030032, China; ^2^Tongji Hospital, Tongji Medical College, Huazhong University of Science and Technology, Wuhan 430030, China; ^3^Department of Lymphoma, Shanxi Bethune Hospital, Shanxi Academy of Medical Sciences Tongji Shanxi Hospital, Third Hospital of Shanxi Medical University, Taiyuan 030032, China

## Abstract

**Objective:**

LCZ696 (sacubitril/valsartan) is an angiotensin II (Ang II) type 1 receptor-neprilysin inhibitor, with effects of immunosuppression, anti-inflammation, antiapoptosis, and antioxidation. The present study was aimed at determining whether LCZ696 has a protective effect against isoproterenol-induced acute heart failure (AHF) in rats.

**Methods:**

SD rats were randomly divided into four groups: control group, HF group, LCZ696 group, and enalapril group. The cardiac function of rats was evaluated using echocardiographic parameters, heart weight (HW), serum levels of cardiac troponin I (cTnI), and lactate dehydrogenase (LDH). HE is staining, which was used to determine the pathological damage of rat myocardial tissue. Also, we measured oxidative stress markers including reactive oxygen species (ROS), malondialdehyde (MDA), superoxide dismutase (SOD), and catalase (CAT). Finally, the expression of Nrf2 signaling pathway-related proteins was determined using Western blot.

**Results:**

Compared with the HF group, LCZ696 could significantly improve cardiac function and myocardial injury in rats and reduce AHF-induced oxidative stress. In addition, the results of Western blot confirmed that LCZ696 could upregulate the expression of Nrf2 and HO-1 while decreasing Keap1 expression.

**Conclusion:**

LCZ696 ameliorates isoproterenol-induced AHF in rats by alleviating oxidative stress injury and activating the Nrf2 signaling pathway.

## 1. Introduction

Heart failure (HF) is a clinical syndrome, in which cardiac functional and/or structural abnormalities lead to impaired ventricular filling or ejection of blood [1]. Acute heart failure (AHF) is an acute exacerbation of preexisting symptoms and signs of HF, and it has become one of the main reasons for hospitalization in patients over 65 years with a high mortality rate [2–3]. Every year, a huge sum of money is spent on the treatment and management of AHF all over the world, and this sum has been increasing in recent years [4]. According to a population survey, 1% to 2% of people aged over 70 are expected to suffer from AHF, and this number will continue to increase by 10% per year [5]. Therefore, it is necessary to explain the pathogenesis of AHF and explore its therapeutic target to effectively minimize the degree of myocardial injury and AHF-caused mortality and improve the prognosis and quality of life of patients.

HF is the terminal stage of a variety of etiologies, and among them, myocardial cell loss is the major contributor to HF [6]. Several studies have found that oxidative stress plays a critical role in apoptosis and is closely involved in the progression of HF [7]. Tissue ischemia and hypoxia severely damage myocardial cells, leading to a decrease in oxidative phosphorylation, a conversion of polyunsaturated fatty acids to lipid peroxides, and an oxidation-antioxidant imbalance and resulting in oxidative stress response. Endogenous catalytic free radicals such as SOD and GSH-Px can convert polyunsaturated fatty acids into nontoxicants or increase their water solubility, therefore exerting antioxidant effects [8]. A study have confirmed that nuclear factor E2-related factor 2 (Nrf2) is a key regulator of redox homeostasis and cellular antioxidant defense. Under steady-state conditions, Nrf2 is immobilized in the cytoplasm by Kelch-like ECH-associated protein 1 (Keap1), a homologous protein that links Nrf2 to the E3 ligase complex [9]. By contrast, when exposed to external stimuli and the oxidative stress is activated, Nrf2 is isolated from the Keap1 and E3 ligase complexes and then translocate to the nucleus [10]. Nrf2 can interact with the phase II antioxidant enzymes, such as HO-1, NQO-1, and has a protective effect on cardiovascular diseases such as atherosclerosis and HF [11].

LCZ696 (sacubitril/valsartan) is an angiotensin II (Ang II) type 1 receptor-neprilysin inhibitor consisting of valsartan and sacubitril and is a preparation that inhibits the root mean square deviation (RMS) while activating the natriuretic peptide system [12]. In recent years, with the deepening of research, its pharmacological activity has also continuously been excavated. The LCZ696 blocks the Ang II receptor and inhibits the release of Ang II-dependent aldosterone through valsartan, thus antagonizing the renin-angiotensin-aldosterone system (RAAS). This in turn reduces sympathetic excitability and myocardial oxygen consumption, improves hemodynamics, inhibits myocardial fibrosis, and therefore slows the development of HF [13]. In contrast, LCZ696 inhibits the degradation of the natriuretic peptide system by neprilysin through sacubitril, thereby enhancing this system. LCZ696 has been proven in animal studies to enhance cardiac function in rats and rabbits with HF by increasing early angiogenesis, enhancing myocardial perfusion, and minimizing myocardial remodeling in rats and rabbits with HF. A small number of domestic studies have revealed that LCZ696 can improve postoperative cardiac function in patients with acute anterior ST-segment elevation myocardial infarction and HF [14–16]. Additionally, the recent studies have reported that LCZ696 can significantly inhibit oxidative stress injury caused by cardiovascular and cerebrovascular diseases [17, 18]. Based on all the above studies, it was hypothesized that LCZ696 improves HF through Nrf2/HO-1 signaling pathway. The present study might play a role to open a new direction and to provide new ideas for the treatment of this disease.

## 2. Materials and Methods

### 2.1. Experimental Animals and Treatment

Twelve-week-old healthy male SD rats weighing 220 ± 30 g with ambient temperature 22 ± 1°C. The rats were allowed to adapt in under a photoperiod of 12 : 12 hour light-dark period. The above rats were randomly divided into four groups: control group, HF group, LCZ696 group, and enalapril group. In the control and HF groups, rats took normal saline orally per day for two consecutive weeks. Rats in the LCZ696 group were treated orally with LCZ696 (68 mg/kg/day), while those in the enalapril group received enalapril orally (20 mg/kg/day). From the second week of administration, rats in the HF, LCZ696, and enalapril groups were intraperitoneally injected with isoproterenol (5 mg/kg) every 24 h for 7 consecutive days to induce rats' models of AHF. Note that rats in the control group were intraperitoneally injected with the same amount of normal saline. The specific process is shown in Figure 1. The animal experiments described in this study were approved by the Ethical Committee of the Shanxi Bethune Hospital.

### 2.2. Echocardiography and Hemodynamic Measurements

After 2 weeks of administration, the rats were anesthetized and placed in the left lateral decubitus position for echocardiography. Left ventricular end-systolic pressure (LVESP), left ventricular end-diastolic pressure (LVEDP), and ejection fraction (EF) were obtained by direct measurement of the long-axis view of the left ventricle.

At the end of the ultrasound, hemodynamic measurements were performed while the rats were kept under anesthesia. The maximum rate of rising of left ventricular pressure (+ dp/dtmax) and the maximum rate of decrease of left ventricular pressure (-dp/dtmax) was recorded. Each index was measured three times, and the results were averaged [19].

### 2.3. Specimen Collection

Rats were anesthetized and sacrificed. Then, blood was collected in heparin tubes and centrifugated at 3000 r/min for 10 min. The supernatant was collected in the Eppendorf tubes (EP tubes). The thoracic cavity was aseptically cut open, and then, myocardial tissue was taken and washed with sterile saline. After the solution on the tissue surface was absorbed by filter paper, a part of the myocardium was fixed in paraformaldehyde for H&E staining, and the other part was stored at -80°C in a screw cap tube for Western blot assay.

### 2.4. Ventricular Mass Index (HW/BW)

Rats were anesthetized and sacrificed. Then, the hearts were immediately removed and placed in precooled normal saline for repeated rinsing to remove residual blood. After that, the atria, great vessels, and epicardial adipose tissue were removed. The hearts were dried with filter paper and weighed with an electronic balance to calculate the ratio of heart weight (HW) to body weight (BW).

### 2.5. Hematoxylin and Eosin Staining

Hematoxylin and Eosin (H&E) was carried out to observe the pathological process of myocardial tissues. First, the tissues were fixed, followed by paraffin embedding and preparation of 4 *μ*m sections. Second, the sections were routinely dewaxed with xylene 3 times, 15, 10, and 10 min each time. Third, the sections were hydrated using gradient ethanol from high concentration to low concentration (100% ethanol I and II for 10 min each; 90% ethanol for 10 min; 80% ethanol for 10 min), followed by water washing thoroughly. Forth, the sections were stained in hematoxylin for 5 min and then rinsed with tap water. Fifth, hydrochloric acid ethanol was used for differentiation for 30 s. Sixth, the sections were immersed in tap water for 15 min. After immersion, eosin solution was adopted for staining for 2 min. The final step was conventional dehydration, clearing, and mounting. The pathological damage of myocardial tissue was observed in the control, HF, LCZ696, and enalapril groups.

### 2.6. Detection of Oxidative Stress Markers and Myocardial Injury Indicators

Myocardial tissues were collected from each group and centrifuged at 3000 r/min for 10 min to obtain supernatant. The activities of reactive oxygen species (ROS), malondialdehyde (MDA), superoxide dismutase (SOD), catalase (CAT), and lactate dehydrogenase (LDH) were measured according to the kit (Solarbio, Beijing, China) instructions and were expressed as U/mL “or U/L.” The content of cardiac troponin I (cTnI) was detected according to the ELISA kit instructions and expressed as pg/mL.

### 2.7. Western Blot

RIPA lysate was used to extract total protein from myocardial tissues. The concentration of total protein was determined by BCA, and the final concentration of protein in each group was adjusted to the same level. SDS-PAGE was then used to separate protein, with specific steps of preparing to separate gel and stacking gel, loading samples, and running the electrophoresis. The separated protein was then transferred to the PVDF membrane, followed by 2 h blocking in TBST buffer containing 5% skimmed milk. Subsequently, the samples were incubated with primary antibodies for 2 h and then incubated with primary antibodies Nrf2 rabbit polyclonal antibody (ab92946, 1 : 1000), HO-1 rabbit monoclonal antibody (ab68477, 1 : 1000), Keap1 mouse monoclonal antibody (ab119403, 1 : 1000), and GAPDH rabbit monoclonal antibody (ab181602, 1 : 1000) overnight at 4°C. The next day, the secondary antibodies labeled with horseradish peroxidase (HRP) were added for 2 h incubation. The color was developed by chemiluminescence, and the results were analyzed by the gel imaging system. Images were subsequently quantified with ImageJ (National Institutes of Health).

### 2.8. Statistical Analysis

The data obtained from the above experiments were statistically analyzed using SPSS 22.0 software. The measured data were expressed as mean ± standard deviation (x ± s). Differences between two groups were compared using a student *t*-test, while those among three groups were compared using a One-Way ANOVA. Each experiment was repeated at least 3 times. The *p* < 0.05 was considered statistically significant.

## 3. Results

### 3.1. Effects of LCZ696 on Hemodynamics and Cardiac Function in Rats with Heart Failure

Compared with the control group, the HF group showed significantly decreased levels of left ventricular systolic pressure (LVSP), EF, +dp/dtmax, -dp/dtmax, and increased LVEDP, indicating the cardiac function of HF rats deteriorated. Treatment with LCZ696 or enalapril could markedly improve cardiac function (Figures 2(a)–2(e)). Ventricular mass index measurement revealed that compared with the control group, a significant decrease in BW and increases in HW and HW/BW were found in the HF group. Further, treatment with LCZ696 or enalapril led to a marked increase in BW, a decrease in HW, and ultimately a decreased ratio of HW/BW (Figures 2(f)–2(h)). The above results indicated that LCZ696 treatment improved hemodynamics and cardiac function in HF rats.

### 3.2. LCZ696 Attenuates Myocardial Injury in Rats with Heart Failure

The results of H&E stain showed that the morphology and structure of myocardial tissue were normal, and the arrangement of myocardial fibers was neat in the control group. Before the administration of isoproterenol, there was significantly decreased levels of LVSP and increased LVEDP which indicates that the cardiac function of HF rats was deteriorated. After rat models of HF induced by isoproterenol, cardiac myocytes swelled and necrosed in HF rats, and myocardial fibers were arranged disorderly with a blurred outline. LCZ696 and enalapril could decrease the swelling, abnormal morphology, and necrosis in cardiac myocytes and result in a more neatly arrangement of myocardial fibers (Figure 3(a)).

Subsequently, the contents of cTnI and LDH in rat serum, indicators of myocardial injury, were measured. The findings revealed that the serum levels of cTnI and LDH were significantly increased in the HF group compared with the control group, suggesting myocardial injury in HF rats. Compared with the HF group, the serum levels of cTnI and LDH were significantly decreased in the LCZ696 and enalapril groups (Figures 3(b) and 3(c)). The above results showed that LCZ696 was able to markedly reduce myocardial injury in AHF rats.

### 3.3. Antioxidant Effect of LCZ696 in Rats with Heart Failure

Oxidative stress injury is the most important secondary injury caused by AHF, and improving this injury as much as possible will have a better protective effect on cardiomyocytes [20, 21]. To clarify whether the protective effect of LCZ696 on the myocardium is related to antioxidant effects, we examined the levels of oxidative stress parameters in myocardial tissue. The experimental results showed that the levels of ROS and MDA were significantly increased, and the levels of SOD and CAT were significantly decreased in the myocardial tissue of the HF group compared with the control group. Treatment with LCZ696 and enalapril could decrease the levels of ROS and MDA while increasing the levels of SOD and CAT in myocardial tissue (Figures 4(a)–4(d)). Taken together, LCZ696 had a good antioxidant effect on HF-induced myocardial injury.

### 3.4. LCZ696 Activates the Nrf2 Signaling Pathway in the Myocardium of Rats with Heart Failure

Numerous studies have shown that the Nrf2 signaling pathway plays an important role in oxidative stress injury [22, 23]. Whether LCZ696 was able to exert antioxidant effects by mediating this pathway was further explored in this study. Western blot was therefore used to detect the expression of Nrf2 signaling pathway-related proteins in myocardial tissue from HF rats. Compared with the control group, Keap1 expression was significantly increased while HO-1 expression was significantly decreased in the myocardial tissue of the HF group. Further, Keap1 expression was lower while HO-1 expression was higher in myocardial tissues of the LCZ696 and enalapril groups compared with the HF group (Figures 5(a) and 5(b)). Additionally, Nrf2 expression in the nucleus was significantly reduced in the myocardial tissue of the HF group, but treatment with LCZ696 and enalapril markedly increased its expression (Figures 5(c) and 5(d)). According to the findings, LCZ696 could activate the Nrf2 signaling pathway in the myocardium of HF rats.

## 4. Discussion

In the current study, the isoproterenol was used to stimulate rat models of AHL and then investigated the protective effects of LCZ696 on the models. Initially, it was found by echocardiography and cardiac anatomy that LCZ696 could improve cardiac function and symptoms of myocardial hypertrophy in HF rats. Secondly, HE stains and serum cTnI and LDH were used to evaluate the pathological damage of myocardial tissue in rats, which confirmed that LCZ696 significantly reduced myocardial injury in HF rats. Thirdly, the antioxidant effect of LCZ696 was then revealed by detecting ROS, MDA, SOD, and CAT levels in rat myocardial tissue. Since the Nrf2 signaling pathway plays a critical role in oxidative stress injury induced by AHF, the expression of Nrf2 signaling pathway-related proteins (Nrf2, HO-1, and Keap1) was also detected by Western blot in this study; LCZ696 was found to promote the translocation of Nrf2 into the nucleus and upregulate the expression of Keap1 and HO-1 genes, thereby reducing oxidative stress and protecting cardiomyocytes. Collectively, the above results indicate that LCZ696 can improve cardiac function by activating the Nrf2 signaling pathway and ultimately inhibits the development of HF. Similar findings were obtained by a recent study in which they treated the DOX-rats using LCZ696. The conducted study concluded that the LCZ696 ameliorated DOC-induced cardiotoxicity in rats' heart *in-vivo* and *in-vitro* could possibly decrease in oxidative stress [24].

The mechanism of myocardial injury caused by HF is not clear. A generally accepted hypothesis suggested that HF-induced oxidative stress is one of the vital triggers leading to injury [25–27]. HF induces a massive generation of ROS by interfering with the normal function of the mitochondrial electron transport chain during oxidative phosphorylation [28]. Our study also found that HF induced ROS accumulation in the rat heart. Excessive ROS induces lipid peroxidation by attacking biofilms, resulting in a significant increase in MDA content in myocardial tissue. Lipid peroxidation can change the physicochemical properties and structure of lipids and interfere with the biological function of lipids. In this study, treatment with LCZ696 could significantly decrease the levels of ROS and MDA in the myocardial tissue of HF rats. Specifically, the experimental results showed that LCZ696 alleviated HF-induced oxidative stress by scavenging ROS and inhibiting lipid peroxidation. To protect cells from ROS damage, the body has a well-established endogenous antioxidant defense system, mainly including antioxidant enzymes and nonenzymatic antioxidants. Antioxidant enzymes such as SOD and CAT have been considered the first line of defense against free radical damage [29, 30]. SOD converts superoxide anion to hydrogen peroxide, and CAT further converts hydrogen peroxide to water [31]. Previously, a study has reported that HF not only induces the production of ROS but exacerbates oxidative stress by disrupting the body's endogenous antioxidant system [32]. Our study found that in the activities of antioxidant enzyme SOD, CAT was significantly decreased in the myocardial tissues of HF rat models, while pretreatment with LCZ696 could significantly increase their activities. These results suggest that the regulation of the endogenous antioxidant defense system by LCZ696 is important in protecting rats from HF-induced myocardial injury. Isoproterenol is widely used to treat heart failure in mice [33]. In the case of chronic heart disease, the SD rats can be pretreated with isoprenaline followed by treating with LCZ6969. The finding would not be same. There is a possibility that both treatments could lead to over oxidative stress.

Nrf2 is a stress-regulated transcription factor. Exposed to both endogenous and exogenous stress, it regulates the expression of antioxidant defense genes (e.g., HO-1, Keap1, and NQO1) by binding to antioxidant response elements in promoter regions [34, 35]. Nrf2 is highly sensitive to the development of common cardiovascular diseases, such as atherosclerosis, hypertension, and diabetic cardiomyopathy; activation of Nrf2 can protect the heart from ischemia-reperfusion injury and inhibit the progression of diabetic cardiomyopathy [36–38]. It has been shown that decreased intercellular ROS and MDA levels and increased SOD and CAT levels contribute to the activation of Nrf2 and play a protective role by inducing its targeted antioxidant genes [39]. One of the most important targets of Nrf2 in endothelial cell homeostasis is HO-1 which usually parallels the upregulation of ferritin to reduce free iron levels and prevent Fenton-like reactions [40]. HO-1 expression in patients with peripheral arterial disease mostly showed a decreasing trend [41]. Previous studies have found by constructing a cardiomyopathy model that the mediation of Nrf2 inhibits the process of isoproterenol-induced cardiomyopathy development, further indicating that the Nrf2/HO-1 signaling pathway is involved in the regulatory process of cardiac injury [42]. Previously, LCZ696 has been proved to inhibit the production of ROS and activate the Nrf2 signaling pathway in cardiomyocytes, thus exerting antioxidative stress, anti-inflammatory, and antifibrosis effects on cardiomyocytes [43]. In this study, a Western blot was used to detect the expression of Nrf2, HO-1, and Keap1, thus further verifying the mechanism of LCZ696. The results revealed that after treatment with LCZ696, Nrf2 expression in the nucleus increased significantly whereas it dramatically decreased in the cytoplasm. We also discovered that following modelling, the protein expression of the above genes was considerably reduced, but the Nrf2/HO-1 signaling pathway was stimulated by administration of LCZ696.

## 5. Conclusion

In summary, LCZ696 can significantly improve cardiac function and hypertrophy, reduce myocardial injury and oxidative stress injury induced by AHF, upregulate Nrf2 and HO-1 expression, and downregulate Keap1 in AHF rats. Therefore, it is unclear that inhibition of Nrf2 translocation could reverse the protective effect of LCZ696 on heart failure. However, further systematic research is crucial to probe the mechanism and regulating Nrf2 signaling pathway, which could still need to be verified by carrying out subsequent animal experiments and collecting clinical tissue samples. Future studies in this field is worthy of systematic in-depth study, thus providing more clinical treatment ideas for cardiovascular diseases such as AHF and an experimental basis for relevant drug research and development.

## Figures and Tables

**Figure 1:** Flow diagram of animal modeling of the current study. The illustration is followed be the previously conducted study [13].

**Figure 2:** Effects of LCZ696 on hemodynamics and cardiac function in rats with heart failure. (*p* = 0.05^∗^ and *p* = 0.01^∗∗^ vs control vs HF). (a) LVESP: Left ventricular end-systolic pressure; (b) LVEDP: Left ventricular end-diastolic pressure; (c) LVEF: Left ventricular ejection fraction; (d) + dp/dtmax, maximum rate of rise of left ventricular pressure; (e) -dp/dtmax, maximum rate of decrease of left ventricular pressure; (f) HW: Heart weight; (g) BW: Body weight; (h) HW/BW. *p* = 0.05^∗^ and *p* = 0.01^∗∗^ vs control; *p* = 0.01^##^ vs HF.

**Figure 3:** Effects of LCZ696 on myocardial injury in rats with heart failure (a) HE staining-based detection of morphology and structure of cardiac myocytes. (b) Serum level of cardiac troponin I (cTnI). (c) Serum level of lactate dehydrogenase (LDH). (*p* = 0.01^∗∗^ vs control; *p* = 0.01^##^ vs HF).

**Figure 4:** Detection of reactive oxygen species (ROS) (a), malondialdehyde (MDA) (b), superoxide dismutase (SOD) (c), and catalase (CAT) (d) in myocardial tissue. (*p* = 0.01^∗∗^ vs control; *p* = 0.01^##^ vs HF).

**Figure 5:** Detection of Nrf2 signaling pathway-related proteins in myocardial tissue by Western blot. (*p* = 0.01^∗∗^ vs control; *p* = 0.01^##^ vs HF).

## Data Availability

The data used to support the findings of this study are available from the corresponding author upon request.

## References

[1] Zsilinszka R., Mentz R. J., DeVore A. D., Eapen Z. J., Pang P. S., Hernandez A. F. (2017). Acute heart failure: alternatives to hospitalization. *Jacc Heart Failure*.

[2] Long B., Koyfman A., Gottlieb M. (2019). Diagnosis of acute heart failure in the emergency department: an evidence-based review. *The Western Journal of Emergency Medicine*.

[3] Ponikowski P., Voors A. A., Anker S. D. (2016). 2016 ESC guidelines for the diagnosis and treatment of acute and chronic heart failure. *Kardiologia Polska*.

[4] Mebazaa A., Tolppanen H., Mueller C. (2016). Acute heart failure and cardiogenic shock: a multidisciplinary practical guidance. *Intensive Care Medicine*.

[5] Dunlay S. M., Roger V. L., Redfield M. M. (2017). Epidemiology of heart failure with preserved ejection fraction. *Nature Reviews Cardiology*.

[6] Hou N., Huang Y., Cai S. A. (2021). Puerarin ameliorated pressure overload-induced cardiac hypertrophy in ovariectomized rats through activation of the PPAR*α*/PGC-1 pathway. *Acta Pharmacologica Sinica*.

[7] Chi J., Li Z., Hong X. (2018). Inhalation of hydrogen attenuates progression of chronic heart failure via suppression of oxidative stress and P 53 related to apoptosis pathway in rats. *Frontiers in Physiology*.

[8] Khan S., Zhang D., Zhang Y., Li M., Wang C. (2016). Wogonin attenuates diabetic cardiomyopathy through its anti-inflammatory and anti-oxidative properties. *Molecular and cellular endocrinology*.

[9] Suzuki T., Yamamoto M. (2015). Molecular basis of the Keap1-Nrf2 system. *Free Radical Biology and Medicine*.

[10] Alfredo S., Maldonado P. D. (2018). Canonical and non-canonical mechanisms of Nrf2 activation. *Pharmacological Research*.

[11] Chen Q. M., Maltagliati A. J. (2018). Nrf2 at the heart of oxidative stress and cardiac protection. *Physiological Genomics*.

[12] Schoenfeld H. A., West T., Verghese P. B. (2017). The effect of angiotensin receptor neprilysin inhibitor, sacubitril/valsartan, on central nervous system amyloid-*β* concentrations and clearance in the cynomolgus monkey. *Toxicology and applied pharmacology*.

[13] Miyoshi T., Nakamura K., Miura D. (2019). Effect of LCZ696, a dual angiotensin receptor neprilysin inhibitor, on isoproterenol-induced cardiac hypertrophy, fibrosis, and hemodynamic change in rats. *Cardiology Journal*.

[14] Ishii M., Kaikita K., Sato K. (2017). Cardioprotective effects of LCZ696 (sacubitril/valsartan) after experimental acute myocardial infarction. *Jacc Basic to Translational Science*.

[15] Xia Y., Chen Z., Chen A. (2017). A metabolomics approach to profiling the cardioprotective effect of LCZ696, an angiotensin receptor-neprilysin inhibitor, on ischemia induced heart failure. *RSC Advances*.

[16] Ushijima K., Ando H., Arakawa Y. (2017). Prevention against renal damage in rats with subtotal nephrectomy by sacubitril/valsartan (LCZ696), a dual-acting angiotensin receptor-neprilysin inhibitor. *Pharmacology Research & Perspectives*.

[17] Mohany M., Alanazi A. Z., Alqahtani F., Belali O. M., Ahmed M. M., al-Rejaie S. S. (2020). LCZ696 mitigates diabetic-induced nephropathy through inhibiting oxidative stress, NF-*κ*B mediated inflammation and glomerulosclerosis in rats. *PeerJ*.

[18] Suematsu Y., Jing W., Nunes A. (2018). LCZ696 (sacubitril/valsartan), an angiotensin-receptor neprilysin inhibitor, attenuates cardiac hypertrophy, fibrosis, and vasculopathy in a rat model of chronic kidney disease. *Journal of Cardiac Failure*.

[19] Zhao Z. Q., Morris C. D., Budde J. M. (2003). Inhibition of myocardial apoptosis reduces infarct size and improves regional contractile dysfunction during reperfusion. *Cardiovascular Research*.

[20] Bergamini C., Cicoira M., Rossi A., Vassanelli C. (2009). Oxidative stress and hyperuricaemia: pathophysiology, clinical relevance, and therapeutic implications in chronic heart failure. *European Journal of Heart Failure*.

[21] Nickel A. G., Von Hardenberg A., Hohl M. (2015). Reversal of mitochondrial transhydrogenase causes oxidative stress in heart failure. *Cell Metabolism*.

[22] Loboda A., Damulewicz M., Pyza E., Jozkowicz A., Dulak J. (2016). Role of Nrf2/HO-1 system in development, oxidative stress response and diseases: an evolutionarily conserved mechanism. *Cellular and molecular life sciences*.

[23] Ueda K., Ueyama T., Yoshida K. I. (2008). Adaptive HNE-Nrf2-HO-1 pathway against oxidative stress is associated with acute gastric mucosal lesions. *AJP Gastrointestinal and Liver Physiology*.

[24] Chang S. C., Ren S., Rau C. D., Wang J. J. (2018). Isoproterenol-Induced Heart Failure Mouse Model Using Osmotic Pump Implantation. *Experimental Models of Cardiovascular Diseases*.

[25] Chen Q. M., Morrissy S., Alpert J. S. (2018). Oxidative Stress and Heart Failure☆. *Comprehensive Toxicology (Third Edition)*.

[26] Koba S., Angiotensin I. I. (2018). Angiotensin II, Oxidative stress, and sympathetic nervous system hyperactivity in heart failure. *Yonago Acta Medica*.

[27] Li J., Ding H., Li Y. (2021). Alarin alleviated cardiac fibrosis via attenuating oxidative stress in heart failure rats. *Amino Acids*.

[28] Han Y., Shi Z., Zhang F. (2014). Reactive oxygen species in the paraventricular nucleus mediate the cardiac sympathetic afferent reflex in chronic heart failure rats. *European Journal of Heart Failure*.

[29] Guan P., Liang Y., Wang N. (2018). Fasudil alleviates pressure overload-induced heart failure by activating Nrf2-mediated antioxidant responses. *Journal of Cellular Biochemistry*.

[30] Martinez P. F., Bonomo C., Guizoni D. M. (2015). Influence of N-acetylcysteine on oxidative stress in slow-twitch soleus muscle of heart failure rats. *Cellular Physiology & Biochemistry*.

[31] Buyuklu M., Kandemir F. M., Set T. (2017). Beneficial effects of ozone therapy on oxidative stress, cardiac functions and clinical findings in patients with heart failure reduced ejection fraction. *Cardiovascular Toxicology*.

[32] Shah A. (2015). Parsing the role of NADPH oxidase enzymes and reactive oxygen species in heart failure. *Circulation*.

[33] Miyoshi T., Nakamura K., Amioka N. (2022). LCZ696 ameliorates doxorubicin-induced cardiomyocyte toxicity in rats. *Scientific Reports*.

[34] Kensler T. W., Wakabayashi N., Biswal S. (2007). Cell survival responses to environmental stresses via the Keap 1-Nrf2-ARE pathway. *Annual review of pharmacology and toxicology*.

[35] Johnson J. A., Johnson D. A., Kraft A. D. (2008). The Nrf2–ARE pathway: an indicator and modulator of oxidative stress in neurodegeneration. *Annals of the New York Academy of Sciences*.

[36] Mimura J., Itoh K. (2015). Role of Nrf2 in the pathogenesis of atherosclerosis. *Free Radical Biology & Medicine*.

[37] Vaziri N. (2012). Protective effect of Nrf2 and catalase in maternal diabetes-induced perinatal hypertension and kidney disease. *Diabetes*.

[38] Gu J., Cheng Y., Wu H. (2017). Metallothionein is downstream of Nrf2 and partially mediates sulforaphane prevention of diabetic cardiomyopathy. *Diabetes*.

[39] Wang Z., Liang M., Li H. (2019). l-Methionine activates Nrf2-ARE pathway to induce endogenous antioxidant activity for depressing ROS-derived oxidative stress in growing rats. *Journal of the Science of Food and Agriculture*.

[40] Kawaguchi K., Lambein F., Kusama-Eguchi K. (2012). Vascular insult accompanied by overexpressed heme oxygenase-1 as a pathophysiological mechanism in experimental neurolathyrism with hind-leg paraparesis. *Biochemical and Biophysical Research Communications*.

[41] Yang X. J., Liu F., Feng N. (2020). Berberine attenuates cholesterol accumulation in macrophage foam cells by suppressing AP-1 activity and activation of the Nrf2/HO-1 pathway. *Journal of Cardiovascular Pharmacology*.

[42] Hasan R., Lasker S., Hasan A. (2020). Canagliflozin attenuates isoprenaline-induced cardiac oxidative stress by stimulating multiple antioxidant and anti-inflammatory signaling pathways. *Scientific Reports*.

[43] Jing W., Vaziri N. D., Nunes A. (2017). LCZ696 (Sacubitril/valsartan) ameliorates oxidative stress, inflammation, fibrosis and improves renal function beyond angiotensin receptor blockade in CKD. *American Journal of Translational Research*.

